The article "Analysis of the Application Effect of Multidisciplinary Team Cooperation Model in Chronic Heart Failure under WeChat Platform" was retracted in 2023. Reasons: signs of a paper mill; suspected computer-generated content; unreliable results or conclusions; concerns about the data.

# Analysis of the Application Effect of Multidisciplinary Team Cooperation Model in Chronic Heart Failure under WeChat Platform

**DOI:** 10.1155/2022/4051955

**Published:** 2022-08-25

**Authors:** Jieyu Huang, Yu Su, Xiucai Mao

**Affiliations:** ^1^Department of Cardiovascular Medicine, Hezhou People's Hospital, Second Ward, Hezhou, China; ^2^Department of Nephrology, Hezhou People's Hospital, Hezhou, China; ^3^Hezhou People's Hospital Nursing Department, Hezhou, China

## Abstract

**Methods:**

From April 2020 to May 2021, 56 patients with CHF who were discharged from the cardiology department of our hospital after treatment were randomly divided into two groups: experimental group (*n* = 28) and control group (*n* = 28). The control group was given conventional nursing measures and health education and discharge instructions, while the experimental group received collaborative multidisciplinary team nursing care based on the WeChat platform on the basis of the control group, all for 3 months. All enrolled patients underwent the Self-Care of Heart Failure Index Version 6.2 (SCHFI v6.2), the Minnesota Living with Heart Failure Questionnaire (MLHFQ), and the 6-minute walking test (6MWT test). The SCHFI v6.2 and MLHFQ scores, 6 MWT test results, and readmission rates within 3 months were observed and compared between the two groups.

**Results:**

There was no significant difference between the SCHFIv6.2 and MLHFQ scores of the two patients at admission and at discharge, and the scores of the experimental group were significantly higher than the scores of the control group at the end of 3 months after discharge. On the other hand, the SCHFIv6.2 and MLHFQ scores of the two groups were significantly higher at discharge compared to admission; the 6-minute walking distance of the experimental group was significantly higher than that of the control group at the end of 3 months. The readmission rate in the experimental group was significantly lower than that in the control group.

**Conclusion:**

The multidisciplinary teamwork model based on the WeChat platform can significantly improve the self-care ability and quality of life of CHF patients and reduce the readmission rate.

## 1. Introduction

Chronic heart failure (CHF) has become a public health problem of global concern, affecting approximately 1% to 2% of the world's population. It poses a serious threat to patients' health, reduces their ability to work and quality of life, and consequently consumes enormous medical resources, and places a heavy burden on families and society [1, 2]. CHF refers to a persistent state of heart failure. The main symptoms are dyspnoea, ankle swelling, fatigue, signs of elevated jugular pressure, lung rale, and peripheral oedema. The current treatment of heart failure includes general, pharmacological, and nonpharmacological treatments, which have reduced the rate of sudden death and improved clinical symptoms in patients with CHF [3, 4], whereas, although clinical treatment can control symptoms quickly, there are many adverse drug reactions such as electrolyte disorders and drug resistance. Furthermore, the goal of CHF treatment is not only to improve symptoms and hospital outcomes, but also to reduce mortality and readmission rates [5]. Thus, patients need to follow not only standardised medication, but also self-care behaviours that focus on various aspects of diet, activity, physical status monitoring, behavioural and emotional management, proper recognition of symptoms, and assessment of treatment effectiveness.

The article "Analysis of the Application Effect of Multidisciplinary Team Cooperation Model in Chronic Heart Failure under WeChat Platform" was retracted in 2023. Reasons: signs of a paper mill; suspected computer-generated content; unreliable results or conclusions; concerns about the data.

Domestic and international studies have shown that a patient-centred, multidisciplinary team-based service model that provides comprehensive and individualised treatment, care, and rehabilitation for patients can improve patient self-management and quality of life and can reduce the number of patient readmissions [6, 7]. However, such multidisciplinary collaborative teams involve more people, are more affected by time and space, and are difficult to organise and implement at a fixed time, in a fixed hospital, or in the community [8]. At present, WeChat, as a rising and rapidly developing mobile new media force, has the advantages of low cost, strong interaction, featured consultation, and intelligent customization of public platform functions, which can penetrate scientific healthcare concepts into people's social circles and social groups, and provide personalized health management services [9–11]. Given the above research base, we believe that the WeChat platform can provide an ideal virtual space for collaborative multidisciplinary interventions to overcome the difficulties in implementing real-life home interventions for patients with CHF, and is important for improving patients' self-care behaviours, improving care outcomes, and reducing the number of patient readmissions. From April 2020 to May 2021, a 3-month multidisciplinary collaborative team-directed intervention study was implemented on 56 patients with stable CHF via the WeChat platform to observe the clinical value of its evaluation on patients, which is reported below.

### 1.1. Study Subjects

A convenience sampling method was used to select 56 patients who were admitted to the cardiology department of our hospital from April 2020 to May 2021 and were diagnosed with CHF as the study population. Diagnostic criteria: meeting the criteria of the guidelines for the diagnosis and treatment of CHF [12]. Diagnostic criteria for cardiac function classification refer to the 1994 New York Heart Association (NY-HA) classification criteria [13]. Inclusion criteria: those who meet the western diagnostic criteria for CHF with class II-III cardiac function; age 18–75 years; systolic insufficiency with left ventricular ejection fraction (LVEF) ≤ 50% on echocardiography; those who sign the informed consent form; the clinical data of the patients was complete. Exclusion criteria: heart failure due to failure of vital organs such as the liver and kidneys; women who are pregnant or lactating, have severe skin infections or are particularly sensitive to certain drugs; patients with severe primary diseases of the liver, kidneys, endocrine system, and haematopoietic system; patients with psychiatric abnormalities and unwillingness to cooperate; patients with factors that increase mortality, such as cardiogenic shock, severe ventricular arrhythmias, complete atrioventricular block, obstructive cardiomyopathy, unrepaired valve disease, constrictive pericarditis, pericardial tamponade, pulmonary embolism, and uncontrolled hypertension (hypertensive crisis, etc.). Fifty-six patients who met the relevant diagnostic and inclusion criteria were divided into experimental and control groups using a random number table. During the study period, there was 1 case of shedding in the control group and no shedding in the experimental group. 28 patients in the experimental group, 15 males and 13 females, age 58–76 years, mean (68.56 ± 5.28) years; cardiac function status: 14 cases of class II, 10 cases of class III, and 4 cases of class IV. In the control group, there were 27 cases, 13 males and 14 females, age 60–78 years, mean (68.45 ± 5.33) years; cardiac function status: class II 15 cases, class III 9 cases, and class IV 3 cases.

The article "Analysis of the Application Effect of Multidisciplinary Team Cooperation Model in Chronic Heart Failure under WeChat Platform" was retracted in 2023. Reasons: signs of a paper mill; suspected computer-generated content; unreliable results or conclusions; concerns about the data.

### 1.2. Case Shedding Criteria

Those who failed to complete the whole study process due to nonchanges in the disease or other reasons; those who received other treatments that may affect the results and affected the later evaluation; and those who experienced deterioration of the disease or other serious complications during the study period that required urgent treatment.

## 2. Study Methods

### 2.1. Intervention Methods

Six experienced cardiology nurses with solid professional knowledge were responsible for case management and all had worked in the specialty for more than one year, with a college degree or above and nurse practitioner or above titles. The research team, based on an extensive literature review, combined with the practical work experience of the group members in CHF diagnosis and management nursing, prepared a CHF nursing instruction manual, including knowledge related to CHF disease, knowledge of medication management, home oxygen therapy, breathing techniques, exercise training, and management of acute exacerbation period.

### 2.2. Control Group

Patients were given systematic CHF treatment in accordance with their medical characteristics and the CHF Treatment Guidelines. In the control group, the nurse in charge of the patient was given an admission education after admission, and during the hospital stay, the patient was given routine nursing measures and health education, including guidance on diet, medication, lifestyle adjustment, regular follow-up, and other routine knowledge, and at the time of discharge, the patient was given routine discharge instructions, and a personalized discharge plan was formulated according to the patient's specific situation. Patients received discharge health education, the content of which was mainly individualised according to the patient's specific mastery of self-management content and practical problems, and patients were encouraged to give feedback after discharge. Patients were followed up by telephone within 1 week after discharge. To reinforce and consolidate the relevant knowledge and skills in the CHF Nursing Manual, to help patients to answer their questions and encourage them to self-manage.

### 2.3. Experimental Group

On the basis of the control group, a multidisciplinary teamwork based on the WeChat platform was implemented to guide the patients to self-manage at home. The intervention period was 3 months. Briefly, a CHF multidisciplinary collaborative guided intervention WeChat group was established with the head nurse of the cardiology department as the group leader and members including the patient, 2 cardiovascular physicians, 6 cardiology nurses, 1 rehabilitation physiotherapist, 1 nutritionist, and 1 psychological counsellor. Responsibilities and division of labour: cardiologists were responsible for comprehensive assessment of patients' conditions, formulation of disease diagnosis and treatment, and management plans; nurses were case managers, each responsible for 5 patients, and established personal WeChat contact with patients. In addition to sending WeChat educational content to patients, they were also responsible for reminding patients to take their medication on time through WeChat, guiding patients to adhere to medical advice, writing the name, method of administration and effect of medication on the medication box, and not to stop taking medication on their own or missing medication. For some patients with poor memory and missed doses, patients were advised to use reminders such as alarm clocks, reminder cards or links to important events or objects in their daily lives to urge them to take their medication on time. In addition, patients were educated to recognise early symptoms such as occult oedema, reduced activity endurance, increased exertional dyspnoea, increased peripheral oedema, or a resting heart rate that was 15–20 beats/min faster than usual and to consult a doctor promptly in order to control the progression of the disease. The rehabilitation physiotherapist was responsible for setting rehabilitation goals and rehabilitation programmes, formulating individualised exercise programmes according to the classification of cardiac function, and encouraging patients to exercise appropriately. For patients in cardiac function class IV, the nurse instructed bedside physical activities and bedside sitting up exercises; for patients in cardiac function class III, they were given bedside chair training and bedside walking assistance; for patients with class II cardiac function, they were instructed to train ward aisle walking, walking, and stair walking, to gradually increase the amount of exercise, all without exertion, and to control their heart rate to 110 beats/min or less after activity, after discharge from hospital, they were instructed to take appropriate exercises such as jogging, cycling, and soft gymnastics, and gradually transition to general physical activities. In addition, we should avoid inducement, prevent upper respiratory tract infection caused by catching cold to aggravate heart failure, maintain emotional stability, avoid fatigue, defecated regularly, keep defecation unobstructed, do not hold breath and exert too much force during defecation, so as not to lead to heart failure, aggravation, or even sudden death. The dietitian assessed the patient's nutritional status, formulated a nutritional support plan, and teached the patient and family to use a beer cap or coke cap and measuring cup for salt and water and to use <5 g/d of salt for cardiac function class II, <2.5 g/d for cardiac function class III, and <1 g/d for cardiac function class IV, or to avoid salt. If taking diuretics, excessive salt restriction in the diet was not necessary. The dietitian also provided a list of common foods that contained water so that patients could calculate their daily intake, provided a list of common foods to facilitate the calculation of daily water intake, and instructed the patient to eat a light and easily digestible diet rich in high quality protein and vitamins. The psychological counsellor provided regular psychological counselling to patients, guided them in self-regulation and emotional control, actively assisted them to participate in the appropriate medical insurance so that they had sufficient expenses to ensure smooth treatment, conducted psychological assessment of patients, provided targeted psychological care for patients, and at the same time encouraged family members to communicate more with patients. Reduced the patient's anxiety and helped him/her to build up the confidence to overcome the disease. On the other hand, the nurse, as a case manager, sent a piece of knowledge and linked about CHF disease to the patients under her charge through WeChat every week. The content was more detailed and comprehensive than the CHF nursing instruction manual, which was discussed and formulated by the team. The case management nurses collected the information separately, and after the team consultant physician had reviewed and agreed, the case management nurses operated and sent it, and the nurse manager implemented supervision of the pushing process. The push was sent in the form of text, pictures, videos, or voice messages, and was sent at a fixed time, once a week for 3 months. Patients were followed up through phone twice a week to solve their problems and difficulties.

The article "Analysis of the Application Effect of Multidisciplinary Team Cooperation Model in Chronic Heart Failure under WeChat Platform" was retracted in 2023. Reasons: signs of a paper mill; suspected computer-generated content; unreliable results or conclusions; concerns about the data.

### 2.4. Observation Indicators

#### 2.4.1. Patient's Ability to Care for Themselves

Self-Care of Heart Failure Index Version 6.2 (SCHFI v6.2). This scale was developed by Riegel et al. [14], based on the Self-Management Scale. The scale consists of 22 items in 3 dimensions: self-care maintenance (10 items), self-care management (6 items), and self-care confidence (6 items), using a 4-point Likert scale with a total score of 22 to 88, with higher scores indicating better self-care status of the patient.

#### 2.4.2. Patient Quality of Life

The Minnesota Heart Failure Quality of Life Questionnaire (MLHFQ) [15]was used to assess patients' quality of life using this scale. The scale includes physical, fatigue, emotional, and economic aspects, with 21 entries, using a Likert 6-point scale with a total score of 105. The assessment time was between 5 and 10 min. Higher scores indicated a poorer quality of life for the patient.

#### 2.4.3. 6MWT

The main objective was to measure the distance of a 6-minute walk, which was an important indicator of objective assessment of cardiac function in patients with CHF. Each patient was picked up by a case management nurse at discharge and at the end of 3 months to the unit where the 6MWT test was performed under medical supervision. The evaluation was performed according to the 2002 American Thoracic Society (ATS) guidelines for the application of the 6-minute walk test [16]. Evaluation criteria: in 1993 Bittner classified the results of the 6MWT into 4 levels according to the condition: level 1 < 300 m, level 2 300–375 m, level 3 375–450 m, and level 4 > 450 m, with lower levels indicating poorer cardiopulmonary function. Termination criteria: the experiment was terminated by the presence of any of the following: chest pain, dyspnoea, lower limb cramps, pallor, etc. [17].

The article "Analysis of the Application Effect of Multidisciplinary Team Cooperation Model in Chronic Heart Failure under WeChat Platform" was retracted in 2023. Reasons: signs of a paper mill; suspected computer-generated content; unreliable results or conclusions; concerns about the data.

#### 2.4.4. Readmission Rate

This was the incidence of rehospitalisation for exacerbation of preexisting disease in the same patient after discharge from hospital. Patients who were hospitalised within 3 months of discharge for exacerbation of chronic heart failure for any reason were considered to have been readmitted. Excluding hospital admissions for surgical conditions, a rehospitalisation within 7 days of discharge was considered a single hospitalisation for the same patient.

### 2.5. Data Collection Methods

Prior to the survey, the first author of this study provided uniform training to the investigators. The SCHFIv6.2 and MLHFQ scales were administered one-to-one with patients' consent at admission, at discharge and 3 months after discharge, respectively; patients' readmission rates were counted 3 months after discharge. Patients were assisted to complete the questionnaire without the use of suggestive words.

### 2.6. Statistical Methods

All data were analysed using SPSS 19.0 statistical software. Measures were expressed by *t*-test and statistical analysis by *χ*^2^ test.

## 3. Results

### 3.1. General Information Comparison

When comparing the baseline data of patients in the experimental and control groups, the differences in age, gender, 6MWT, NY-HA cardiac function classification, and BNP levels were not statistically significant (*P* > 0.05) and were comparable; see Table 1.

### 3.2. Comparison of Self-Care Capabilities

There was no significant difference between the SCHFIv6.2 scores of the two patients at admission and at discharge, and at the end of 3 months after discharge, the scores in the experimental group were significantly higher than those in the control group. At the end of 3 months after discharge, the experimental group scores were significantly higher than the scores at discharge; however, the control group scores were lower than at discharge (Table 2).

### 3.3. Quality of Life Comparison

There was no significant difference between the MLHFQ scores of the two patients at admission and discharge, and the scores of the experimental group were significantly higher than the scores of the control group at the end of 3 months after discharge. At the end of 3 months postdischarge, the scores in the experimental group were significantly higher than the scores at discharge; however, the scores in the control group were lower than at discharge (Table 3).

The article "Analysis of the Application Effect of Multidisciplinary Team Cooperation Model in Chronic Heart Failure under WeChat Platform" was retracted in 2023. Reasons: signs of a paper mill; suspected computer-generated content; unreliable results or conclusions; concerns about the data.

### 3.4. 6MWT Distance Comparison

The difference in 6MWT between the two groups at admission and discharge was not statistically significant. At the end of 3 months, 6MWT was (471.32 ± 32.43) *m* in the experimental group and (215.41 ± 22.56) *m* in the control group, excluding one case of termination of the experiment due to angina pectoris. The results showed that at the end of 3 months after discharge, the difference in 6MWT between the two groups was statistically significant, with the experimental group significantly higher than the control group. See Table 4.

### 3.5. Comparison of Readmission Rates

The readmission rate within 3 months was 14.28% (4 cases) in the experimental group and 44.45% (12 cases) in the control group. The results showed that the readmission rate in the experimental group was significantly lower than that in the control group, and the difference was statistically significant. Among them, one case in the experimental group was lower than two cases in the control group for rehospitalisation caused by improper medication; three cases in the experimental group were lower than nine cases in the control group for rehospitalisation caused by improper life management (infection, exertion, and diet). For details, see Table 5.

## 4. Discussion

CHF has become a serious public health problem worldwide, and epidemiological data in recent years has reported that the prevalence of heart failure in China is 0.9%, with 4.5 million patients suffering from heart failure and about 500,000 new cases of heart failure each year [18–20]. Various end-stage cardiac diseases can lead to heart failure to varying degrees, including coronary heart disease, hypertension, arrhythmias, heart valve disease, and cardiomyopathy. Of these, coronary artery disease and hypertension account for the highest proportion [21]. The multidisciplinary collaborative model has become the more respected model of CHF management in national and international academia [1, 22, 23]. The current multidisciplinary model of CHF is mainly implemented during the patient's hospitalisation, and it is difficult to organise a multidisciplinary team to provide comprehensive and individualised care and rehabilitation after the patient is discharged from the hospital [24–26]. With the popularity of smartphones, the WeChat platform as a new mobile media has its own advantages in the prevention and treatment of chronic diseases, such as large amount of information, wide coverage; wide range of users, rapid dissemination; peer-to-peer communication, personalized mutual assistance; and multimedia communication, low cost [10, 27, 28]. The WeChat platform is a good solution to the problem of inconsistency in time and place, and team members can communicate with each other and collaborate in multiple disciplines in the virtual network of WeChat [29]. China's chronic disease self-management WeChat intervention projects focus on diabetes, coronary heart disease, hemodialysis, chronic hepatitis, chronic obstructive pulmonary disease, etc. [30, 31], there is less research on self-management WeChat intervention for CHF patients. This study attempted to realize the multidisciplinary cooperation of CHF through WeChat platform and guided patients to carry out family self-management through point-to-many and point-to-point methods. The research results showed that patients had high recognition for the multidisciplinary collaborative team intervention mode based on WeChat platform.

The article "Analysis of the Application Effect of Multidisciplinary Team Cooperation Model in Chronic Heart Failure under WeChat Platform" was retracted in 2023. Reasons: signs of a paper mill; suspected computer-generated content; unreliable results or conclusions; concerns about the data.

There is a widely accepted concept in academia that “self-management is the best option for chronic disease management” [32]. However, it has been reported that ≤7% of people with chronic diseases are actually self-managing worldwide. The vast majority of patients have difficulty with the question of how to self-manage their chronic disease [33]. This study addressed this substantial issue by conducting a self-management intervention guided by a multidisciplinary facilitated team via a WeChat platform in patients with stable CHF. It was found that the multidisciplinary collaborative team intervention based on the WeChat platform all significantly improved the self-management ability of stable CHF patients and patients' quality of life, which may be related to the fact that the multidisciplinary collaborative team intervention increased patients' awareness of the disease to enhance their self-management compliance and helped them to develop good rehabilitation behaviours. In addition, after 3 months of the WeChat-based multidisciplinary team intervention, the patients' knowledge of the specialty and the 6-minute walking distance markedly improved.

According to statistics, the readmission rate of CHF patients is 24.8% within 30 d after discharge and 67.4% within 1 year [34, 35]. Reducing hospital readmissions for CHF patients has become an urgent issue for countries around the world [36–38]. A research has proved that multidisciplinary collaboration is effective in reducing readmission rates for CHF patients [39]. In the current study, we found that the patients in the experimental group, under the dynamic observation and continuous supervision of the case management nurses over a period of 3 months, mastered the adverse effects of the drugs they were taking and the importance of adhering to them, their own dietary structure, and specific intake; learned to arrange their work and rest schedules and exercise reasonably; and gradually improved their ability to manage themselves out of the hospital and their quality of life, resulting in a significant reduction in readmission rates.

The article "Analysis of the Application Effect of Multidisciplinary Team Cooperation Model in Chronic Heart Failure under WeChat Platform" was retracted in 2023. Reasons: signs of a paper mill; suspected computer-generated content; unreliable results or conclusions; concerns about the data.

Patients with severe heart, lung and kidney disease, cardiogenic shock, severe ventricular arrhythmias, complete atrioventricular block, obstructive cardiomyopathy, unrepaired valvular disease, constrictive pericarditis, pericardial tamponade, pulmonary embolism, and uncontrolled hypertension (hypertensive crisis, etc.) were excluded from this study. Therefore, the sample size was small and a larger sample would have been included in the study.

## 5. Conclusion

In summary, despite the improving treatment modalities for CHF, the readmission rate for patients with CHF remains high. A collaborative multidisciplinary team model based on the WeChat platform has been used in a study to reduce readmission of CHF patients, with the intervention providers being predominantly nurse practitioners and multidisciplinary teams. A discharge plan is developed for patients with CHF who are predischarged from the hospital. Postdischarge patients are given multidisciplinary guidance on medication, diet, health, and psychological guidance, and enhanced management through a microsoft platform with real-time follow-up and feedback. Strengthening medication comparison and carrying out remote monitoring are conducive to facilitating timely and continuous care services for CHF patients during their transition from hospital to home, improving patients' self-management and quality of life, and reducing readmission rates.

## Figures and Tables

**Table 1:** Comparison of baseline information between the two groups of patients [$\bar{\chi }\pm S$, (*n*, %)].

Groups	*n*	Age	Gender (*n*, *χ*^2^)		6MWT	Classification of cardiac function			BNP
		(year $\bar{\chi }\pm S$)	Male	Female	(*m*, $\bar{\chi }\pm S$)	II	III	IV	(pg/ml, $\bar{\chi }\pm S$)
Experimental group	28	68.56 ± 5.28	15	13	195.46 ± 20.13	14	10	4	342.13 ± 282.14
Control group	27	68.45 ± 5.33	13	14	196.52 ± 21.36	15	9	3	350.46 ± 267.25
Statistical values	—	0.078^*a*^	0.162^*b*^		0.191^*a*^	0.212^*b*^			0.113^*a*^
*p*-value	—	0.938	0.687		0.849	0.899			0.910

*Note.* ^*a*^ is the value of *t* and ^*b*^ is the value of *χ*^2^. *P* < 0.05 means the difference is statistically significant.

**Table 2:** Comparison of SCHFIv6.2 scores between the two groups of patients $\left(\bar{\chi }\pm S\right)$.

Groups	*n*	On admission	On discharge from hospital	At the end of 3 months after discharge from hospital
Experimental group	28	33.45 ± 4.65	54.23 ± 5.87	60.14 ± 5.84
Control group	27	33.56 ± 3.98	54.12 ± 5.23	50.47 ± 6.23
*t*-value	—	0.095	0.074	5.992
*p*-value	—	0.924	0.941	0.000

*Note. P* < 0.05 means the difference is statistically significant.

The article "Analysis of the Application Effect of Multidisciplinary Team Cooperation Model in Chronic Heart Failure under WeChat Platform" was retracted in 2023. Reasons: signs of a paper mill; suspected computer-generated content; unreliable results or conclusions; concerns about the data.

**Table 3:** Comparison of MLHFQ scores between the two groups $\left(\bar{\chi }\pm S\right)$.

Groups	*n*	On admission	On discharge from hospital	At the end of 3 months after discharge from hospital
Experimental group	28	75.65 ± 6.58	55.42 ± 4.73	45.23 ± 3.85
Control group	27	74.81 ± 6.84	54.65 ± 5.21	55.24 ± 4.74
*t*-value	—	0.089	0.579	8.674
*p*-value	—	0.929	0.565	0.000

*Note. P* < 0.05 means the difference is statistically significant.

**Table 4:** Comparison of 6MWT distances between the two groups of patients $\left(\bar{\chi }\pm S\right)$.

Groups	*n*	On admission	On discharge from hospital	At the end of 3 months after discharge from hospital
Experimental group	28	195.46 ± 20.13	250.45 ± 22.47	471.32 ± 32.43
Control group	27	196.52 ± 21.36	251.32 ± 23.14	215.41 ± 22.56
*t*-value	—	0.191^*a*^	0.143	34.278
*p*-value	—	0.849	0.887	0.000

*Note. P* < 0.05 means the difference is statistically significant.

**Table 5:** Comparison of readmission rates between the two groups within 3 months of discharge (*n*, %).

Groups	*N*	Rehospitalisation	Reason for rehospitalisation	
			Improper administration of medication	Inappropriate diet and lifestyle habits
Experimental group	28	4 (14.28)	1 (3.57)	3 (10.71)
Control group	27	12 (44.45)	2 (7.14)	9 (32.14)
*χ* ^2^- value	—	0.014	—	—
*p*-value	—	0.030	—	—

*Note. P* < 0.05 means the difference is statistically significant.

## Data Availability

The datasets used and analysed during the current study are available from the corresponding author upon reasonable request.
